This article has been retracted.

# Paeoniflorin Attenuated TREM-1-Mediated Inflammation in THP-1 Cells

**DOI:** 10.1155/2022/7051643

**Published:** 2022-04-18

**Authors:** Li Cao, Kerong Yang

**Affiliations:** ^1^Department of Critical Medicine, Shenzhen Baoan Shiyan People's Hospital, Shenzhen 5515108, China; ^2^Department of Suzhou Medical College, Soochow University, Suzhou 215123, China

## Abstract

Sepsis is caused by bacterial infections or viral infections. Clinically, there exist confirmed or highly suspected infection foci. Mortality caused by septic shock remains in a high rate even though antibiotic treatment works effectively. In this study, we treat THP-1 cells with 1 ug/mL LPS (lipopolysaccharide) and add paeoniflorin or LR-12 inhibitor. TREM-1 (triggering receptor expressed on myeloid cells-1), IL-6, IL-1*β*, and TNF-*α* (tumour necrosis factor alpha (a)-cachectin) were detected by ELISA and qRT-PCR, and western blotting is performed to detect related proteins in the NF-*κ*B signaling pathway. As a result, paeoniflorin can significantly reduce the production of LPS-stimulated TREM-1 as well as inflammatory factors and attenuate the phosphorylation of NF-*κ*B signaling pathway-related factors, such as p65 and I*κ*B*α*. At the same time, the combined effect of paeoniflorin and LR-12 is more significant. The results of this study solidly prove that paeoniflorin plays a role in inhibiting TREM-1-mediated inflammation and the NF-*κ*B pathway could be a potential mechanism of action.

## 1. Introduction

Sepsis originates from the complex interaction between infected microorganisms and host immune inflammation [1]. Inflammatory responses are triggered by bacterial pathogens and their products through activated transcription of inflammatory genes, triggering a huge number of relevant mediators released. On the one hand, inflammatory mediators can protect the host from bacteria invading; on the other hand, cells and tissues are also damaged by these mediators. Multiple organ dysfunction syndrome (MODS) represents the most common cause of death in the intensive care unit (ICU) in the 1990s. MODS is characterized by a complex and overwhelming host response involving immune, metabolic, neuroendocrine, and inflammatory mechanisms that usually occurs after massive injury or infection. MODS could be an exemplification to illustrate how uncontrolled or excessive, mediators could damage the body. Despite advances in drug therapy has been made, sepsis-induced MODS is still one of the main cause of death in clinical patients, especially in intensive care units (ICUs) [2]. In the last decade, even though the mortality rate of sepsis has decreased, 29-30% of patients with severe sepsis still die, notably who suffered septic shock reached 60% of mortality [3, 4]. Therefore, MODS remains a major challenge for doctors worldwide [5].

Paeoniflorin is the main bioactive ingredient extracted from *Paeonia lactiflora*. It has pharmacological effects, such as antihyperglycemia [6], anti-inflammatory [7], liver protection [8], cognitive enhancement [9], neuroprotection [10, 11], and antineoplastic [12] properties. Studies [13] showed that paeoniflorin can reduce inflammatory factors in serum of experimental sepsis model mice, and the levels of myeloperoxidase was also reduced in several internal organs, such as lung, liver, and small intestine. Furthermore, paeoniflorin was found to reduce BLP-induced inflammation in THP-1 cells via inhibiting NF-*κ*B signal transduction [14]. Nevertheless, the anti-inflammatory theory of paeoniflorin remains obscure and need further evaluation.

TREM-1 serves as an amplifier, and neutrophils, monocytes, macrophages, and endothelial cells are account for its expression, of which responsible for inflammatory response [15]. As a membrane-bound receptor, TREM-1 is present in human body fluids in a measurable soluble form (sTREM-1). It has been proved that sTREM-1 level works as an indicator for early diagnosis and prognostic marker for part of infectious diseases. A case in point is that sTREM-1 level has been found elevated in bronchoalveolar sac fluid in patients with bacterial pneumonia [16]. In addition, take lipopolysaccharide (LPS) induction experiment for example. TREM-1 consumption reduces systemic cytokine production and improves survival in acute lung injury mice [17]. In addition, TREM-1 silencing and response blocking were proven to inhibit cytokines production, such as IL-1*β*, TNF-*α*, and IL-6, and prolong sepsis mice survival [18–21]. Altogether, the above studies support that TREM-1 accounts for inflammatory response and that inflammatory response could be alleviated by interfering it.

In this paper, we illustrate that TREM-1-mediated inflammation is attenuated by paeoniflorin in THP-1 cells and further verified the NF-*κ*B pathway involved in the mechanism.

## 2. Western Blot and Enzyme-Linked Immunosorbent Assay

### 2.1. Cell Culture

THP-1 macrophages (human) are frozen in our laboratory. It requires RPMI-1640 containing 10% FBS (Gibco, Inc.) and 100 U/mL penicillin, at 37°C in an incubator with 5% CO2. Besides, 1 *μ*g/ml of LPS alone was needed for stimulation of THP-1 (LPS group). At the same time, an increasing dose (10^−8^, 10^−6^, and 10^−4^ M) of paeoniflorin (L + 10^−8^ PE, L + 10^−6^ PE, L + 10^−4^ PE group) or 25 *μ*g/ml LR-12 as the L + LR-12 group is administrated, respectively.

### 2.2. CCK-8

Cell Counting Kit-8 (Transgen, China) detects cell viability. First, THP-1 is dispersed at a density of 0.5 × 10^4^ and inoculated in 96-well plates, and then incubated with medium containing paeoniflorin (0, 10^−8^ M, 10^−6^ M, 10^−4^ M, or 10^−2^ M) for 24 h. Second, CCK-8 agents (10 ul) and serum free 1640 medium (90 ul) are added, and the plates are further incubated for 2 h. Finally, 450 nm absorbance will be read and used to do the cell viability calculation. Three independent experiments are needed for each sample.

### 2.3. TUNEL

24-well plates are used for THP-1 seeding, with 1 × 10^6^ cells per well and exposed to the indicated treatments. Then, TUNEL analysis is used to assess cell scorching. First, 4% paraformaldehyde is used for THP-1 cells fixation. Second, 0.1% Triton X-100 was used for cells permeabilization. Next, TUNEL reaction mixture with cells at 37°C will be left in the dark for 1 hour. Finally, after 15 minutes of DAPI staining, confocal laser scanning microscopy detects the cell fluorescence.

### 2.4. Real-Time Quantitative PCR Analysis

Trizol reagent (Invitrogen) for RNA extraction can be applied. First, PrimerScript RT reagent Kit (Takara) is used for first-strand cDNA synthesization. Then, SYBR Premix Ex Taq (Takara Bio) for quantify the amount of mRNA of the interested genes and GAPDH in ABI one-step plus system.  Table 1 demonstrates the primer information for amplification procedure.

### 2.5. Western Blot

Protease and phosphatase inhibitors are indispensable, and total protein will be extracted using RIPA (CWBIO, China) and determined by the BCA protein assay (Beyotime, China). Then, the extracted proteins are analysed using electrophoresis on SDS-polyacrylamide gel. After that, the proteins are transferred to nitrocellulose membrane (Millipore, Ireland). Blocking process was performed by skim milk; then, the proteins with the primary antibody were kept overnight at 4°C, cleaned, and will be followed by the secondary antibody incubation at room temperature for 1 hour each. Western blotting was performed using Pierce Biotechnology. The applied antibodies are p-p65, p-I*κ*B*α*, and *β*-actin (Abcam). The signals are quantified and visualized by using the ImageJ software.

### 2.6. Enzyme-Linked Immunosorbent Assay

TNF-*α*, IL-6, and IL-1*β* of THP-1 are detected by the relevant ELISA kit (BYabscience, China). Three independent experiments will be performed. Data were analyzed by using the SPSS v21.0 software. Statistical significance is confirmed by Student's *t*-test. *P* < 0.05 indicates significance.

## 3. Result

### 3.1. Paeoniflorin Alters LPS-Upregulated TREM-1

Firstly, we employed CCK-8 to measure the cell viability of THP-1 under the gradient incubation of paeoniflorin concentration for 24 h. The results show that when paeoniflorin concentration was less than 10^−4^ M, the cell survival rate was over 90%, and the cell viability was decreased at 10^−2^ M dose of paeoniflorin, as shown in Figure 1(a). Therefore, the concentrations in subsequent experiments are 10^−8^ M, 10^−6^ M, and 10^−4^ M, respectively. The qRT-PCR results show that the mRNA level of TREM-1, at the time point of 24 h, was significantly increased under LPS treatment compared with the control group. However, paeoniflorin could effectively inhibit LPS-upregulated TREM-1 mRNA expression in a concentration-related way, as shown in Figure 1(b). Similarly, sTREM-1 in cell supernatant is observed by ELISA and performs a consistent trend, as shown in Figure 1(c). TUNEL shows that LPS increased the apoptosis rate of THP-1, but the addition of paeoniflorin does not further induce apoptosis, as shown in Figures 1(d) and 1(e). These results suggest that paeoniflorin can significantly inhibit LPS-upregulated TREM-1 expression in THP-1.

### 3.2. Paeoniflorin Affects LPS-Stimulated Proinflammatory Cytokines

At the same time, proinflammatory cytokine levels are monitored at 24 h. LPS treatment notably increases TNF-*α*, IL-1*β*, and IL-6 expression in THP-1. It is evidenced by ELISA results, which is shown in Figures 2(a)–2(c). The addition of paeoniflorin inhibited the increase of LPS-stimulated consequence. Furthermore, the intensifying inhibitory effect will be triggered by exposing cells to the increased paeoniflorin concentration. Similarly, as shown in Figures 2(d)–2(f), those proinflammatory cytokines can be detected by qRT-PCR, which also shows a similar trend regarding mRNA levels. These data suggest that paeoniflorin may significantly reduce those cytokines, of which exhibiting an increased tendency in THP-1 through LPS stimulation.

### 3.3. LR-12 Influences LPS-Stimulated TREM-1 and Proinflammatory Cytokines

LR-12 is a known inhibitor of specific TREM-1. We conduct the experiments to obtain the performance of LR-12 with or without paeoniflorin on LPS-induced changes in TREM-1 and cytokine expression levels.  Figure 3 shows the administration of paeoniflorin and LR-12, which resulted in the expression changes of LPS-stimulated TREM-1 and proinflammatory cytokine in THP-1. As can be seen from the result in Figures 3(a) and 3(b), similar to paeoniflorin, LR-12 effectively reduced LPS-stimulated TREM-1 mRNA and the amount of sTREM-1 in the supernatant. As can be seen from Figures 3(c)–3(h), qRT-PCR and ELISA show that LR-12 attenuates those mentioned cytokines. In addition, we also observe from the results that the inhibition effect exhibited more significantly when paeoniflorin and LR-12 were used simultaneously.

### 3.4. Paeoniflorin Impacts LPS-Induced Changes of NF-*κ*B Signaling

Since the NF-*κ*B signaling is closely related with the inflammatory cytokines production, we investigate whether it is associated with the anti-inflammatory effect of paeoniflorin. Thus, to further delineate the impacts of paeoniflorin on THP-1 cells, NF-*κ*B signaling proteins, p-P65, and pI*κ*B*α* are observed. As a result, LPS treatment significantly increases phosphorylation of those proteins.  Figure 4 shows that the paeoniflorin impacts NF-*κ*B signaling-related proteins in THP-1 cells. As can be seen from Figures 4(a)–4(c), paeoniflorin and LR-12 significantly inhibited NF-*κ*B phosphorylation. At the same time, the effect of paeoniflorin combined with LR-12 is more significant.

## 4. Discussion

Septic shock is caused by severe bacterial or viral infection, which can occur unpredictably and can progress rapidly in hospital intensive care units [22, 23]. Despite the availability of effective antibiotics, septic shock still has a high mortality rate [21, 24]. We propose an idea about the role of paeoniflorin in LPS-induced sepsis, focusing on the effect of paeoniflorin on TREM-1-mediated inflammatory response and its mechanism.

Interestingly, soluble form sTREM-1 is simultaneously released [25]. Moreover, many studies have proven that TREM-1 can serve as an effective amplifier for drug proinflammatory responses [18, 26, 27]. An animal study shows that blocking TREM-1 signaling reduced inflammatory mediators and prolonged survival in infected mice [28]. In vitro studies have shown that LPS-stimulated monocyte TREM-1 expression is increased, accompanied by increased cytokine levels [29]. In our study, TREM-1 is significantly upregulated in LPS-stimulated THP-1, accompanied with proinflammatory cytokines upregulation, such as IL-6, IL-1*β*, and TNF-*α*, whereas paeoniflorin could significantly inhibit TREM-1-mediated inflammatory response.

LR-12 is a well-recognized inhibitor of specific TREM-1. It has potent immunomodulatory properties that inhibit the TREM-1 inflammatory amplification loop but do not completely eliminate the inflammatory response [30]. Researchers have found out that continuous intravenous administration of high doses of LR-12 (6 mg/kg/7 h 45 min) in humans remained safe and well tolerated, with few side effects after administration [31]. As an inhibitory peptide of TREM-1, LR-12 has therapeutic effects on a variety of infectious and noninfectious diseases. It has been found that LR-12 can reduce LPS-induced inflammation by modulating the immune response thereby improving survival in mice [32]. Also, in an ape model of LPS-induced sepsis, LR-12 attenuated endotoxin-mediated blood pressure reduction and inflammatory factor release without significant side effects and attenuated endotoxin-related clinical and biological alterations [33]. Furthermore, studies have shown that LR-12 can reduce several proinflammatory cytokines in plasma and improve the survival rate of mice in sepsis model mice [34]. Our study shows that LR-12, like paeoniflorin, significantly delayed the elevation of TREM-1, IL-6, IL-1*β*, and TNF-*α* levels in THP-1. At the same time, the combination of paeoniflorin and LR-12 shows more significant inhibition.

NF-*κ*B is a crucial factor regulating a serial of physiological and pathological processes, where inflammatory factors, such as IL-6, IL-1*β*, and TNF-*α*, are highly involved in the courses [35]. NF-*κ*B signal activation triggers phosphorylation of P65 as well as I*κ*B*α* [36]. Previous studies have shown that the inflammation regulating act of TREM-1, for which the potential mechanism may lie in NF-*κ*B signaling activation [37, 38]. The p-P65 and pI*κ*B*α*-related proteins in NF-*κ*B signaling will be obviously upgraded under LPS stimulation, and the addition of paeoniflorin and LR-12 significantly inhibit the phosphorylation of NF-*κ*B signaling. It suggests that paeoniflorin inhibits TREM-1-mediated reactions via NF-*κ*B signaling.

## 5. Conclusions

Our study illustrates that TREM-1 is a magnifier of SIRS associated with sepsis. It amplifies the inflammatory response in concert with Nod-like and toll-like receptors, promoting the secretion and release of inflammatory factors such as IL-1*β*, IL-8, and TNF-*α* . When stimulated by LPS, TREM-1 upregulation can cause non-negligible consequence with regard to inflammatory process far more obvious than TREM-1 or TLR-4 alone. TREM-1 also upregulates the expression of various adhesion molecules on myeloid cells (such as neutrophils), making them adhere to the matrix and promoting chemotactic migration. Thus, TREM-1 is able to increase the inflammatory response, and overactivation can lead to an uncontrolled expansion of the inflammatory response. In the event of an inflammatory response, inflammatory factors such as IL-6 and TNF-*α* can synergize with the LPS-TLR-4 signaling pathway, thus enhancing TREM-1 production, continuously enhancing such inflammatory response.

Generally, our observations suggest that TREM-1 plays a crucial part upon LPS-stimulated THP-1 inflammation. Paeoniflorin can inhibit the production of TREM-1-mediated cytokines, possibly by disturbing the NF-*κ*B signaling. Therefore, we define a molecular basis for the treatment of bacterial lipoprotein-induced sepsis. In the future, we will make further research of the pharmacology in terms of the paeoniflorin in inhibiting TREM-1-mediated inflammation. In addition, we will conduct more medical experiments to explore the mechanism of NF-*κ*B pathway gradually.

## Figures and Tables

**Figure 1:** Paeoniflorin alters TREM-1 in LPS-stimulated THP-1: (a) CCK-8 detected the effects of paeoniflorin at different concentrations on THP-1; (b) the relative transcription level of TREM-1 mRNA; (c) sTREM-1 of THP-1 was determined by ELISA; (d) the apoptosis of THP-1 induced by LPS and paeoniflorin was detected by TUNEL. ^*∗*^*P* < 0.05, untreated control group; ^#^LPS, *P* < 0.05. L: LPS; PF: paeoniflorin; (e) mean ± SEM.

**Figure 2:** Paeoniflorin affects LPS-induced IL-6, IL-1*β*, and TNF-*α* concentrations in THP-1: (a) TNF-*α*; (b) IL-1*β*; (c) IL-6; (d) relative TNF-*α* expression; (e) relative IL-1*β* expression; and (f) relative IL-6 expression.

**Figure 3:** Administration of paeoniflorin and LR-12 resulted in the expression changes of LPS-stimulated TREM-1 and proinflammatory cytokine in THP-1: (a) sTREM-1; (b) relative TREM-1 expression; (c) TNF-*α*; (d) IL-1*β*; (e) IL-6; (f) relative TNF-*α* expression; (g) relative IL-1*β* expression; and (h) relative IL-6 expression.

**Figure 4:** Paeoniflorin impacts NF-*κ*B signaling-related proteins in THP-1 cells: (a) expression of p-P65 and p-I*κ*B*α* compared with the *β*-actin by western blotting; (b)^*∗*^*P* < 0.05 vs. control group; (c)^#^*P* < 0.05 vs. LPS. ^∧^*P* < 0.05 vs. the L + 10^−4^ PF and L + LR-12 group.

**Table 1:** Primer sequence.

GAPDH	F: 5′-GAAGGTGAAGGTCGGAGTC-3′
	R: 5′-GAAGATGGTGATGGGATTTC-3′

TNF-*α*	F: 5′-CCTCTCTCTAATCAGCCCTCTG-3′
	R: 5′-GAGGACCTGGGAGTAGATGAG-3′

IL-1*β*	F: 5′-TTCGACACATGGGATAACGAGG-3′
	R: 5′-TTTTTGCTGTGAGTCCCGGAG-3′

IL-6	F: 5′-CCTGAACCTTCCAAAGATGGC-3′
	R: 5′-TTCACCAGGCAAGTCTCCTCA-3′

## Data Availability

The simulation experiment data used to support the findings of this study are available from the corresponding author upon request.
